The article "VEGF Genetic Polymorphisms May Contribute to the Risk of Diabetic Nephropathy in Patients with Diabetes Mellitus: A Meta-Analysis" was retracted in 2020. Reasons: errors in the analysis; errors in the results or conclusions; errors in the text; plagiarized text.

# *VEGF* Genetic Polymorphisms May Contribute to the Risk of Diabetic Nephropathy in Patients with Diabetes Mellitus: A Meta-Analysis

**DOI:** 10.1155/2014/624573

**Published:** 2014-08-11

**Authors:** Li Sun, Quan Yuan, Ning Cao, Wei Guo, Li Yao, Jiang-Min Feng, Jian-Fei Ma, Li-Ning Wang

**Affiliations:** ^1^Department of Nephrology, The First Affiliated Hospital of China Medical University, Shenyang 110001, China; ^2^Department of Orthopedics, Shengjing Hospital of China Medical University, Shenyang 110004, China; ^3^Department of Blood Purification, General Hospital of Shenyang Military Region, Shenyang 110015, China; ^4^Department of Nephrology, The Fourth People's Hospital of Shenyang, Shenyang 110034, China

## Abstract

*Objective*. This meta-analysis aimed to investigate a comprehensive and reliable conclusion on the correlations of single nucleotide polymorphisms (SNPs) in the vascular endothelial growth factor (*VEGF*) gene with the risk of diabetic nephropathy (DN) in patients with diabetes mellitus (DM). *Methods*. We screened PubMed, Embase, Web of Science, Cochrane Library, CISCOM, CINAHL, Google Scholar, CBM, and CNKI databases for those relevant studies that investigated the association of 14,945 subjects with clinicopathological parameters in gastric cancer. *Results*. Eleven case-control studies that met all inclusion criteria were included in this meta-analysis. A total of 14,945 subjects were involved, including 3,049 DN patients and 11,896 DM patients. Our meta-analysis results revealed that *VEGF* rs2010963 and rs3025039 polymorphisms might contribute to the risk of DN in DM patients. Ethnicity-stratified analysis suggested that *VEGF* genetic polymorphisms were associated with an increased risk of DN among Asians. However, we found no correlations of *VEGF* genetic polymorphisms with susceptibility to DN among Caucasians. *Conclusion*. Our findings suggest that *VEGF* rs2010963 and rs3025039 polymorphisms may contribute to the risk of DN in DM patients, especially among Asians. Thus, *VEGF* genetic polymorphisms could be useful biomarkers for early diagnosis of DN in DM patients.

## 1. Introduction

Diabetic nephropathy (DN), also identical to intercapillary glomerulonephritis or nodular diabetic glomerulosclerosis, is among the most lethal complications that occur in patients with type 1 or type 2 diabetes mellitus (DM) [1, 2]. It is well known that DN can cause death two or three years after the initial lesions appear; it is more frequent in men and has become a secondary cause of death among end-stage renal diseases [3–5]. In general, DN is a multifactorial disease induced by complex interactions between environmental factors and genetic determinants [6, 7]. Several factors always contributing to DN risk include abnormal renal hemodynamic responses, fatty acid metabolism caused by hyperglycemia, hypertension, and abnormal metabolism of vasoactive substances [8]. Currently, vascular endothelial growth factor (*VEGF*) has also been reported to be associated with the development and progression of DN [9, 10].

The article "VEGF Genetic Polymorphisms May Contribute to the Risk of Diabetic Nephropathy in Patients with Diabetes Mellitus: A Meta-Analysis" was retracted in 2020. Reasons: errors in the analysis; errors in the results or conclusions; errors in the text; plagiarized text.

*VEGF* is a secreted mitogen highly specific for vascular endothelial cells, which have been implicated in endothelial cell proliferation and migration [11]. The human* VEGF* gene is located on chromosome 6p21.3 and composed of 8 exons and 7 introns, with an overall length of approximately 14 kb [12]. As a potent multifunctional cytokine, VEGF has been commonly considered as a prime determinant and regulator of angiogenesis, vasculogenesis, and vascular permeability [13, 14]. A number of epidemiological studies have demonstrated that VEGF plays a crucial role in the pathogenesis of diabetic microvascular complications, including diabetic retinopathy and DN [15–17]. VEGF is responsible for mediating angiogenesis by increasing vascular permeability to water and proteins, while excessive vascular permeability during pathological angiogenesis may contribute to the development and progression of DN [18]. In addition, genetic variations in the* VEGF* gene might lead to high-level expression of* VEGF*. However, high expression of* VEGF* may alter intracellular signal transduction, promote extracellular matrix synthesis, and stimulate renal hypertrophy, which are thought to be key factors in the increase of susceptibility to DN [19, 20]. Therefore, it was postulated that single nucleotide polymorphisms (SNPs) in the* VEGF* gene could be functional and were associated with an increased risk of DN [21]. Abundant studies have indicated that* VEGF* genetic polymorphisms may play an important role in the development of DN [22, 23]. However, results of these studies have been contradictory [24–26]. This meta-analysis was performed to evaluate the relationships of* VEGF* genetic polymorphisms with the risk of DN in DM patients.

## 2. Materials and Methods

### 2.1. Literature Search

Studies addressing the correlations of VEGF genetic polymorphisms with the risk of diabetic nephropathy in patients with diabetes mellitus were identified by searching for articles in the following electronic databases: the Medline (1966~2013), the Cochrane Library Database (Issue 12, 2013), Embase (1980~2013), PubMed (1966~2013), CINAHL (1982~2013), Web of Science (1945~2013), and Chinese Biomedical Database (CBM) (1982~2013). Various combination of keywords and MeSH terms: [“SNP” or “mutation” or “genetic polymorphism” or “variation” or “polymorphism” or “single nucleotide polymorphism” or “variant”] and [“diabetic nephropathies” or “DN” or “diabetic kidney disease”] and [“vascular endothelial growth factors” or “VEGF” or “vascular permeability factor” or “VPF”]. We also performed a manual search of the reference lists from the relevant articles to find other potential articles.

The article "VEGF Genetic Polymorphisms May Contribute to the Risk of Diabetic Nephropathy in Patients with Diabetes Mellitus: A Meta-Analysis" was retracted in 2020. Reasons: errors in the analysis; errors in the results or conclusions; errors in the text; plagiarized text.

### 2.2. Selection Criteria

The eligible studies included in our meta-analysis should meet the following types of inclusion criteria: (1) the study design must be clinical cohort or case-control study; (2) the study must relate to the relationships of* VEGF* genetic polymorphisms with the risk of DN in DM patients; (3) all patients must conform to the diagnostic criteria of DN; (4) the study must provide sufficient information about the frequencies of SNPs. If the study could not meet the inclusion criteria, it would be excluded. The most recent or the largest sample size publication was included when the authors published several studies using the same subjects.

### 2.3. Data Extraction

Two authors from each included study used a standardized form to systematically collect relevant data. The researchers collected the following data: the first author and publication year of article, language of publication, geographical location, design of study, sample size, the source of the subjects, allele frequencies, source of samples, genotyping method of SNP, evidence of Hardy-Weinberg equilibrium (HWE), and so forth.

### 2.4. Quality Assessment

Methodological quality was independently assessed by two researchers according to the Newcastle-Ottawa Scale (NOS) criteria [27]. The NOS criteria included three aspects: (1) subject selection: 0~4; (2) comparability of subject: 0~2; (3) clinical outcome: 0~3. NOS scores ranged from 0 to 9, and a score of  ≥7 indicates a good quality.

### 2.5. Statistical Analysis

The STATA version 12.0 (Stata Corp, College Station, TX, USA) software was used for meta-analysis. We calculated crude odds ratios (ORs) with their 95% confidence intervals (95% CI) to evaluate their relationships under 5 genetic models: the allele model (mutant [M] allele versus wild [W] allele), the dominant model (WM + MM versus WW), the recessive model (MM versus WW + WM), the homozygous model (MM versus WW), and the heterozygous model (MM versus WM). The *Z* test was used to estimate the statistical significance of pooled statistics. The Cochran's* Q*-statistic and *I* ^2^ test were used to evaluate potential heterogeneity between studies [28]. If* Q*-test shows a *P* < 0.05 or *I* ^2^ test exhibits >50% which indicates significant heterogeneity, the random effect model was conducted or else the fixed effects model was used. We also performed subgroup and metaregression analyses to investigate potential sources of heterogeneity. In order to evaluate the influence of single studies on the overall estimate, sensitivity analysis was performed. We conducted Begger's funnel plots and Egger's linear regression test to investigate publication bias [29].

The article "VEGF Genetic Polymorphisms May Contribute to the Risk of Diabetic Nephropathy in Patients with Diabetes Mellitus: A Meta-Analysis" was retracted in 2020. Reasons: errors in the analysis; errors in the results or conclusions; errors in the text; plagiarized text.

## 3. Results

### 3.1. Characteristics of Included Studies

Initially, the searched keywords identified 308 articles. We reviewed the titles and abstracts of all articles and excluded 154 articles; full texts and data integrity were also reviewed and 142 articles were further excluded (Figure 1). Finally, 11 case-control studies were included in this meta-analysis [18, 22–26, 30–34]. Publication years of the eligible studies ranged from 2005 to 2013. The distribution of the number of topic-related literatures in electronic databases during the last decade is shown in Figure 2. A total of 14,945 subjects were involved, including 3,049 DN patients and 11,896 DM patients. Overall, eight studies were conducted among Asians, and three studies were conducted among Caucasians. The classical polymerase chain reaction-restriction fragment length polymorphism (PCR-RELP) method was performed in eight studies, while the other three studies used TaqMan assay, PCR-amplicon sequence analysis (PCR-ASA), and Pyrosequencing methods. The NOS scores of all included studies were ≥5. We summarized the study characteristics and methodological quality in Table 1.

### 3.2. Quantitative Data Synthesis

Meta-analysis findings on the relationships of* VEGF* genetic polymorphisms with the risk of DN in DM patients were shown in Table 2. The random effects model was conducted since significant heterogeneity existed between studies. Our meta-analysis results revealed that* VEGF* rs2010963 (allele model: OR = 1.26, 95% CI = 1.05~1.52, *P* = 0.015; dominant model: OR = 1.29, 95% CI = 1.05~1.59, *P* = 0.015; recessive model: OR = 1.44, 95% CI = 1.00~2.05, *P* = 0.047; homozygous model: OR = 1.65, 95% CI = 1.08~2.50, *P* = 0.020; resp.) and rs3025039 (allele model: OR = 1.38, 95% CI = 1.06~1.80, *P* = 0.018; dominant model: OR = 1.53, 95% CI = 1.02~2.27, *P* = 0.037; homozygous model: OR = 1.56, 95% CI = 1.06~2.30, *P* = 0.023; resp.) polymorphisms might contribute to the risk of DN in DM patients (Figure 3). Nevertheless, no similar associations were found in other polymorphisms in the* VEGF* gene (all *P* > 0.05).

Subgroup analysis by ethnicity suggested that* VEGF* genetic polymorphisms were associated with an increased risk of DN among Asians (allele model: OR = 1.36, 95% CI = 1.17~1.59, *P* < 0.001; dominant model: OR = 1.46, 95% CI = 1.19~1.79, *P* < 0.001; recessive model: OR = 1.46, 95% CI = 1.12~1.91, *P* = 0.005; homozygous model: OR = 1.72, 95% CI = 1.27~2.31, *P* < 0.001; resp.) (Figure 4). However, we found no correlations of* VEGF* genetic polymorphisms with susceptibility to DN among Caucasians (all *P* > 0.05). Further subgroup analysis by genotyping method showed significant associations between* VEGF* genetic polymorphisms and DN risk in the PCR-RFLP subgroup (allele model: OR = 1.31, 95% CI = 1.13~1.52, *P* < 0.001; dominant model: OR = 1.44, 95% CI = 1.21~1.71, *P* < 0.001; recessive model: OR = 1.32, 95% CI = 1.03~1.70, *P* = 0.029; homozygous model: OR = 1.57, 95% CI = 1.18~2.10, *P* = 0.002; resp.) but not in the non-PCR-RFLP subgroup (all *P* > 0.05).

The article "VEGF Genetic Polymorphisms May Contribute to the Risk of Diabetic Nephropathy in Patients with Diabetes Mellitus: A Meta-Analysis" was retracted in 2020. Reasons: errors in the analysis; errors in the results or conclusions; errors in the text; plagiarized text.

Metaregression analysis confirmed that SNP type and ethnicity might be the main sources of heterogeneity (as shown in Table 3). The results of sensitivity analysis suggested that no single study could influence the overall pooled estimates (Figure 5). We found no evidence of obvious asymmetry in the Begger's funnel plots (Figure 6). Egger's test also did not display strong statistical evidence for publication bias (allele mode: *t* = 2.92, *P* = 0.011 and dominant model: *t* = 2.53, *P* = 0.024, resp.).

## 4. Discussion 

VEGF is a potent multifunctional cytokine belonging to the multipotent cytokines family [35]. The role of VEGF has been primarily investigated in its regulation of angiogenesis [9, 18]. It should be noted that VEGF mediates angiogenesis in part by increasing normal vascular permeability to water and proteins [9]. However, excessive vascular permeability during pathological angiogenesis may in turn conduce to macro- or microvascular diseases in some way [18]. Recently, high VEGF concentrations have been detected in patients with respiratory diseases or diabetic microvascular complications including DN, which indicated VEGF might play a major role in the susceptibility to DN [18, 36]. It is widely accepted that VEGF was involved in the induction and maintenance of the fenestrae in glomerular capillary endothelial cells [37, 38], while genetic abnormalities in* VEGF* gene may result in the aberrancy of glomerular filtration barrier and renal tubular reabsorption, which can eventually lead to the occurrence of microalbuminuria and proteinuria [39, 40]. Therefore,* VEGF* genetic variants have been postulated to be clearly an excellent candidate for the pathogenesis of DN [21, 41].

In the present meta-analysis, we evaluated the relationships of* VEGF* genetic polymorphisms with the risk of DN in DM patients. Finally, 11 independent case-control studies were included. Our meta-analysis results showed positive associations of* VEGF* rs2010963 and rs3025039 polymorphisms with susceptibility to DN in DM patients, indicating that these polymorphisms may be causative factors for the incidence of DN. Although the exact function of* VEGF* gene in the development of DN is not fully understood, a potential explanation might be that variants in the* VEGF* gene increased its expression level which was suspected to play a vital role in injury of podocytes by acting in a novel autocrine signaling mode to induce the podocytopathy of diabetes and the genesis of albuminuria related with DN. Our findings were in accordance with a previous study which attempted to show that* VEGF* genetic polymorphisms had a significantly higher frequency in DN patients with microalbuminuria or proteinuria than in DM patients [22]. Since obvious heterogeneity existed, we also performed stratified analysis based on ethnicity and genotyping method. Our results suggested that there was significant correlation of* VEGF* genetic polymorphisms with an increased risk of DN among Asians and the PCR-RFLP subgroup but not among Caucasians and in the non-PCR-RFLP subgroup, which indicated that ethnic differences and genotype may be the main sources of heterogeneity. All in all, our findings were consistent with previous studies that found* VEGF* genetic polymorphisms may alter the risk of developing DN in DM patients, suggesting that these polymorphisms may be utilized as biomarkers for early diagnosis and prognosis of DN.

The article "VEGF Genetic Polymorphisms May Contribute to the Risk of Diabetic Nephropathy in Patients with Diabetes Mellitus: A Meta-Analysis" was retracted in 2020. Reasons: errors in the analysis; errors in the results or conclusions; errors in the text; plagiarized text.

Although this is the first meta-analysis focused on the association of* VEGF* genetic polymorphisms with the risk of DN in DM patients, our study still has some limitations. Firstly, our results had lacked sufficient statistical power to assess the correlations between genetic variants of* VEGF* and susceptibility to DN due to the relatively small sample size. Secondly, meta-analysis is a retrospective study that may lead to subject selection bias, thereby affecting the reliability of our results. Thirdly, our meta-analysis failed to obtain original data from the included studies, which may limit further evaluation of potential roles of* VEGF* genetic polymorphisms in the development and progression of DN. Importantly, the inclusion criteria of cases and controls were not well defined in all included studies, which might also influence our results.

In conclusion, our findings supply convincing evidence that* VEGF* rs2010963 and rs3025039 polymorphisms may contribute to the risk of DN in DM patients, especially among Asians. Thus,* VEGF* genetic polymorphisms could be useful biomarkers for early diagnosis of DN in DM patients. However, due to the limitations mentioned above, more studies with larger sample sizes are still needed to provide a more representative statistical analysis accurately.

The article "VEGF Genetic Polymorphisms May Contribute to the Risk of Diabetic Nephropathy in Patients with Diabetes Mellitus: A Meta-Analysis" was retracted in 2020. Reasons: errors in the analysis; errors in the results or conclusions; errors in the text; plagiarized text.

## Figures and Tables

**Figure 1:** Flow chart of literature search and study selection. Eleven case-control studies were included in this meta-analysis.

**Figure 2:** Distribution of the number of topic-related literatures in the electronic database during the last decade.

**Figure 3:** Forest plots for the relationships of* VEGF* genetic polymorphisms with the risk of diabetic nephropathy in patients with diabetes mellitus under the allele and dominant models.

**Figure 4:** Subgroup analyses by ethnicity of the relationships of* VEGF* genetic polymorphisms with the risk of diabetic nephropathy in patients with diabetes mellitus under the allele and dominant models.

**Figure 5:** Sensitivity analysis of the summary odds ratio coefficients on the relationships of* VEGF* genetic polymorphisms with the risk of diabetic nephropathy in patients with diabetes mellitus under the allele and dominant models.

**Figure 6:** Begger's funnel plot of publication biases on the relationships of* VEGF* genetic polymorphisms with the risk of diabetic nephropathy in patients with diabetes mellitus under the allele and dominant models.

**Table 1:** Baseline characteristics and methodological quality of all included studies.

First author	Year	Country	Ethnicity	Sample size		Gender (M/F)		Age (years)		Genotyping method	SNP type	HWE test (*P* value)	NOS score
				DN	DM	DN	DM	DN	DM				
Bonnefond [18]	2013	France	Caucasian	1510	10581	917/593	6739/3842	64.3 ± 10.0	62.9 ± 10.1	TaqMan	rs6921438 Y/X	0.953	7
									60.4 ± 9.7		rs10738760 Y/X	0.095	
Nikzamir [23]	2012	Iran	Asian	255	235	129/126	106/129	59.6 ± 8.1	58.4 ± 7.6	PCR-RFLP	rs2010963 G/C	0.401	6
Xiao [25]	2011	China	Asian	111	105	63/48	55/50	63.4 ± 6.8	60.5 ± 6.2	PCR-ASA	rs699947 G/A	0.118	7
Zhang [26]	2008	China	Asian	102	92	54/48	44/48	59.9 ± 12.4	61.6 ± 10.4	PCR-RFLP	rs3025039 C/T	0.063	7
Zhang [34]	2008	China	Asian	173	123	—	—	63.7 ± 10.6	62.7 ± 9.9	PCR-RFLP	rs3025039 C/T	0.581	7
Guo [30]	2008	China	Asian	81	76	41/40	35/41	59.6 ± 10.9	57.1 ± 10.9	PCR-RFLP	rs2010963 G/C	0.425	7
											rs833061 C/T	0.172	
Xue [33]	2007	China	Asian	97	60	44/53	29/31	—	65.6 ± 11.6	PCR-RFLP	−2549 D/I	0.368	8
McKnight [22]	2007	UK	Caucasian	242	301	149/93	122/179	17.6 ± 9.0	15.9 ± 8.4	Pyrosequencing	rs3025039 C/T	0.712	7
										TaqMan	rs699947 G/A	0.182	
										Pyrosequencing	rs2010963 G/C	0.055	
Buraczynska [24]	2007	Poland	Caucasian	245	91	126/119	43/48	57.9 ± 10.7	56.9 ± 9.8	PCR-RFLP	−2549 D/I	0.679	8
											rs2010963 G/C	0.652	
He [31]	2007	China	Asian	129	120	64/65	56/64	62.9 ± 12.0	61.6 ± 15.3	PCR-RFLP	rs3025039 C/T	0.661	7
Li [32]	2005	China	Asian	104	112	58/54	50/48	62.1 ± 7.0	60.0 ± 6.8	PCR-RFLP	rs2010963 G/C	0.511	8

DN: diabetic nephropathy; DM: diabetes mellitus; M: male; F: female; SNP: single nucleotide polymorphism; PCR-RFLP: polymerase chain reaction-restriction fragment length polymorphism; PCR-ASA: polymerase chain reaction-amplicon sequence analysis; HWE: Hardy-Weinberg equilibrium; NOS: the Newcastle-Ottawa Scale.

The article "VEGF Genetic Polymorphisms May Contribute to the Risk of Diabetic Nephropathy in Patients with Diabetes Mellitus: A Meta-Analysis" was retracted in 2020. Reasons: errors in the analysis; errors in the results or conclusions; errors in the text; plagiarized text.

**Table 2:** Meta-analysis of the relationships of *VEGF *genetic polymorphisms with the risk of diabetic nephropathy in patients with diabetes mellitus.

	M allele vs. W allele			WM + MM vs. WW			MM vs. WW + WM			MM vs. WW			MM vs. WM		
	(Allele model)			(Dominant model)			(Recessive model)			(Homozygous model)			(Heterozygous model)		
	OR	95% CI	*P *	OR	95% CI	*P *	OR	95% CI	*P *	OR	95% CI	*P *	OR	95% CI	*P *
Overall	1.17	1.05−1.29	0.004	1.20	1.04−1.39	0.010	1.17	1.02−1.34	0.030	1.29	1.06−1.56	0.010	1.12	0.98−1.28	0.103

SNP															
rs6921438 Y/X	0.88	0.76−1.04	0.130	0.83	0.65−1.06	0.129	0.88	0.67−1.16	0.366	0.79	0.58−1.09	0.152	0.94	0.70−1.26	0.682
rs10738760 Y/X	1.08	0.93−1.27	0.316	1.13	0.88−1.45	0.339	1.09	0.84−1.41	0.522	1.16	0.85−1.58	0.337	1.05	0.79−1.38	0.751
rs2010963 G/C	1.26	1.05−1.52	0.015	1.29	1.05−1.59	0.015	1.44	1.00−2.05	0.047	1.65	1.08−2.50	0.020	1.28	0.94−1.74	0.115
rs699947 G/A	1.04	0.85−1.29	0.668	0.95	0.69−1.30	0.736	1.22	0.85−1.75	0.288	1.15	0.75−1.76	0.516	1.29	0.86−1.96	0.223
rs3025039 C/T	1.38	1.06−1.80	0.018	1.53	1.02−2.27	0.037	1.39	0.98−1.98	0.062	1.56	1.06−2.30	0.023	1.27	0.87−1.84	0.210
rs833061 C/T	1.17	0.74−1.83	0.502	1.16	0.59−2.29	0.659	1.42	0.57−3.55	0.449	1.50	0.54−4.16	0.431	1.38	0.53−3.56	0.507
2549 D/I	1.12	0.84−1.50	0.442	1.27	0.84−1.92	0.251	0.98	0.57−1.69	0.951	1.13	0.62−2.08	0.684	0.88	0.50−1.56	0.661

Ethnicity															
Caucasians	1.03	0.95−1.12	0.449	1.02	0.90−1.16	0.711	1.07	0.93−1.23	0.368	1.07	0.91−1.26	0.421	1.07	0.92−1.24	0.401
Asians	1.36	1.17−1.59	<0.001	1.46	1.19−1.79	<0.001	1.46	1.12−1.91	0.005	1.72	1.27−2.31	<0.001	1.31	0.99−1.74	0.061

Method															
Non-PCR-PFLP	1.04	0.94−1.14	0.453	1.00	0.88−1.15	0.944	1.10	0.94−1.28	0.247	1.11	0.90−1.36	0.344	1.10	0.94−1.29	0.232
PCR-RFLP	1.31	1.13−1.52	<0.001	1.44	1.21−1.71	<0.001	1.32	1.03−1.70	0.029	1.57	1.18−2.10	0.002	1.16	0.90−1.51	0.243

W: wild allele; M: mutant allele; WW: wild homozygote; WM: heterozygote; MM: mutant homozygote; OR: odds ratio; 95%CI: 95% confidence interval; SNP: single nucleotide polymorphism.

**Table 3:** Univariate and multivariate metaregression analyses of potential source of heterogeneity.

Heterogeneity factors	Coefficient	SE	*Z *	*P *	95% CI	
					LL	UL
Publication year						
Univariate	−0.349	0.016	−2.21	0.027	−0.066	−0.004
Multivariate	−0.062	0.035	−1.75	0.080	−0.132	0.007
SNP type						
Univariate	−0.063	0.026	−2.43	0.015	−0.113	−0.012
Multivariate	−0.037	0.033	−1.13	0.258	−0.101	0.027
Country						
Univariate	0.031	0.040	0.79	0.431	−0.046	0.108
Multivariate	−0.101	0.080	−1.26	0.206	−0.257	0.055
Ethnicity						
Univariate	0.264	0.088	2.99	0.003	0.091	0.437
Multivariate	0.199	0.088	2.25	0.025	0.025	0.372
Method						
Univariate	−0.222	0.088	−2.52	0.012	−0.395	−0.049
Multivariate	−0.047	0.137	−0.34	0.733	−0.315	0.222

SE: standard error; 95%CI: 95% confidence interval; UL: upper limit; LL: lower limit; SNP: single nucleotide polymorphism.
